This article has been retracted.

# Factors associated with induced abortion in Nepal: data from a nationally representative population-based cross-sectional survey

**DOI:** 10.1186/s12978-019-0732-7

**Published:** 2019-05-28

**Authors:** Suresh Mehata, Jamie Menzel, Navaraj Bhattarai, Sharad Kumar Sharma, Mukta Shah, Erin Pearson, Kathryn Andersen

**Affiliations:** 1 Ipas Nepal, Baluwatar, Nepal, Do Cha Marg, Ward No.: 04, Kathmandu, 44600 Nepal; 2 Ipas, United States, P.O. Box 9990, Chapel Hill, NC 27515 USA; 3 Ministry of Health, Ram Shah Path, Kathmandu, 44600 Nepal

**Keywords:** Abortion, Service utilization, Demographic health survey, Nepal

## Abstract

**Background:**

Despite the legalization of abortion services in 2002, unsafe abortion (abortion services conducted by persons lacking necessary skill or in substandard settings or both) continues to be a public health concern in Nepal. There is a lack of national research exploring the characteristics of women who choose to have an abortion. This study assessed abortion in Nepal and its correlates using data from a nationally representative population-based cross-sectional survey.

**Methods:**

We employed data from the Nepal Demographic and Health Survey 2016. Sample selection was based on stratified two-stage cluster sampling in rural areas and three-stage sampling in urban areas. The primary outcome is report of induced abortion in the 5 years preceding the survey, as recorded in the pregnancy history. All values were weighted by sample weights to provide population-level estimates. Bivariate and multivariate logistic regressions were performed using STATA 14 considering cluster sampling design.

**Results:**

A total of 12,862 women of reproductive age (15–49 years) were interviewed. Overall, 4% (95% CI: 3.41–4.29) reported an abortion within the last 5 years (and less than 1% had had more than one abortion during that time). A higher proportion of women aged 20–34 years (5.7%), women with primary education (5.1%), women aware of abortion legalization (5.5%), and women in the richest wealth quintile (5.4%) had an abortion in the past 5 years. Compared to women aged < 20 years, women aged 20–34 years had higher odds (AOR: 5.54; 95% CI: 2.87–10.72) of having had an abortion in the past 5 years. Women with three or more living children had greater odds (AOR: 2.24; 95% CI: 1.51–3.31) of having had an abortion than women with no living children. The odds of having an abortion in the past 5 years increased with each wealth quintile, with the richest wealth quintile having almost three-fold greater odds of having had an abortion. No significant association was observed between having an abortion and the ecological zone and place of residence.

**Conclusion:**

This nationally representative study shows that abortion is associated with women’s age, knowledge of abortion legality, wealth status, number of living children, and caste/ethnicity. Targeted interventions to young women, those in the poorest wealth quintile, women from Terai caste groups, and those who reside in Province 2 would be instrumental to address disproportional access to abortion services. Overall, strengthening contraceptive provision and abortion education programs would be cornerstone to improving the health of women and girls in Nepal.

## Plain English summary

Unsafe abortion is one of the leading causes of maternal deaths. Many factors contribute to the high prevalence of unsafe abortion in Nepal. Despite the need, limited studies have been conducted on this subject, hence, the findings from this study will be helpful in future program planning and decision making.

This study utilized data from a nationally representative population-based cross-sectional survey to explore the association between induced abortion in Nepal and socio-demographic characteristics, economic status, and knowledge on abortion legalization. A total of 12,862 women of reproductive age were recruited in the study and information was collected using a standard questionnaire which included maternal factors, household-level variables, and community-level variables. To determine the factors associated with abortion, bivariate and multivariate logistic regressions were performed.

The study revealed that abortion was higher among women aged 20–34 compared to aged < 20 years. Compared with women with higher educational levels, women with primary-level education were more likely to have had an abortion. Similarly, women in the richest wealth quintile had a higher likelihood of having an abortion in the last 5 years when compared with those in the poorest wealth quintile. Higher likelihoods of abortion were observed among women who have knowledge of abortion legalization compared to those having no knowledge. A lower proportion of abortion was seen among women who belong to Terai Dalit, Janjatis, and Muslims.

The findings suggest the need to strengthen abortion awareness programs towards youth in the poorest wealth quintile and belonging to specific ethnic groups.

## Background

Worldwide, unsafe abortion is one of the leading causes of and accounts for 7.9% of maternal deaths [1]. Twenty-five million unsafe abortions take place annually and almost all (97%) occur in developing countries [2]. Prior to the legalization of abortion in Nepal, the maternal mortality ratio (MMR) was 850 per 100,000 live births. Up to 20% of these deaths and 54% of obstetric complications were attributable to unsafe abortion [3, 4]. In Nepal, the law permits abortion up to 12 weeks of gestation on request, up to 18 weeks of gestation in cases of rape or incest, and anytime during pregnancy if the woman’s physical/mental health or life is at risk or there is a fetal abnormality that is incompatible with life [5]. Nepal’s abortion policy and service implementation, along with efforts to strengthen antenatal care, emergency obstetrics, and family planning care, have contributed to its impressive 72% reduction in MMR from 850 to an estimated 239 per 100,000 live births between 1991 and 2016 [6]. However, a significant decline is still needed to improve women’s health outcomes and to increase progress toward the Sustainable Development Goals [7]. Despite the liberal abortion law and availability of safe abortion services, unsafe abortion remains a public health concern in Nepal.

Unsafe abortion, defined as termination of an unwanted pregnancy by people lacking the necessary skills or in an environment lacking minimal medical standards or both [2], is the third leading cause of maternal mortality in Nepal, accounting for 7% of maternal deaths [8]. Of an estimated 323,000 abortions performed in Nepal in 2014, only 42% were provided by trained providers in government approved health facilities, and the remaining 58% were considered unsafe [9]. Many factors contribute to the high incidence of unsafe abortion in Nepal. One of the major factors is limited knowledge about the availability of abortion services. According to the Nepal Demographic Health Survey (NDHS) 2016, only 41% of women said they think abortion is legal in Nepal, just a 3% increase from 2011 [10]. Additionally, detailed knowledge of the abortion law and knowledge of where to access safe abortion care is poor [11, 12]. Many socio-cultural barriers and structural factors such as social stigma, limited availability of abortion services, poor quality of abortion services, and economic costs associated with abortion services also restrict women’s access to safe abortion care [13–17].

Although prior studies have explored the association between abortion and other correlates in Nepal, they were mostly limited to a single geographic region, most often from the capital city, Kathmandu, where service access is easy unlike rest of country and socio-economic context is distinct [14, 18]. As a result, the findings from these studies may not be sufficient to represent the entire population. Additionally, there are gaps in the current body of knowledge that explores the correlates of abortion with socio-demographic characteristics, knowledge on legality of abortion, and sex of youngest living child. This study explores correlates of abortion to consider whether Nepali women have equitable access to abortion care.

Many barriers prevent Nepali women from accessing safe abortion services [19, 20]. This often results in women resorting to unsafe abortion and bearing the risk of morbidity/mortality associated with unsafe services [21]. These women are also at a higher risk of having unwanted births [22]. These barriers are multifactorial, including both client-related factors, such as a lack of awareness on abortion legality including legal conditions and availability of services, low economic status, fear of stigma/discrimination, and health system factors, such as poor coverage of health facilities and limited trained providers, especially in rural and hard to reach areas [17, 23]. Both client- and system-related barriers contribute to increased inequality in the utilization of safe abortion services in Nepal.

## Methods

### Data source

This study uses data from the NDHS 2016. A detailed description of the NDHS 2016 methodology and sampling has been described elsewhere [10]. In brief, the sample selection was based on stratified two-stage cluster sampling in rural areas and three-stage sampling in urban areas. First, 383 primary sampling units (wards) were selected with probability proportional to ward size. Subsequently, a fixed number of 30 households per cluster were selected with an equal probability systematic selection. Interviews were completed for 11,040 households, with a response rate of 98.5%. In the interviewed households, 13,089 women of reproductive age (15–49 years) were identified for interviews, and interviews were completed with 12,862 women for a 98.3% response rate [12].

### Variables

The primary outcome of interest was report of an induced abortion in the 5 years preceding the survey. A detailed pregnancy history was collected from women of reproductive age and pregnancy outcomes were categorized as abortion, delivery, miscarriage, or stillbirth, as per the woman’s report. A dichotomous variable was created based on whether any pregnancy ended in an induced abortion within the previous 5 years. To confirm whether the abortion was induced or not, the question was phrased as “Did you or someone else do something to end this pregnancy?” Of the 12,862 women of reproductive age included in the sample, 492 reported 567 pregnancies ending in induced abortion in the last 5 years.

The questionnaire included the following explanatory variables: maternal factors (e.g., age and education), household-level variables (e.g., caste/ethnic group and wealth quintile), and community-level variables (e.g., urban/rural residence, province, and ecological zone). Politically, the country was divided into seven provinces in 2015. The provinces are yet to get their names and are not at an equal level of socio-economic context, including the access to health facilities and care. The method used to compute the wealth index is described in the NHDS 2016 report [10]. In brief, it was derived using principal component analysis, which included information on the number and kinds of consumer goods, such as owning a bicycle or car, and housing characteristics, such as source of drinking water and availability of toilet facilities. Additionally, the number of living children and number of living boy children were included in this analysis. The living boy child variable was created from the birth order questionnaire related to child’s sex and child’s survival status. Knowledge of abortion legality was also used as a predictor variable.

### Statistical analysis

All analyses were performed using STATA 14. Reported values were weighted by sample weights to provide population estimates. Chi-square tests were used to measure the association between the predictor variables and abortion in the last 5 years and adjusted for the survey design, including clustering and urban/rural stratification.

Bivariate logistic regression was used to calculate the unadjusted association of abortion in the last 5 years with each predictor variable. In the adjusted model, multivariate logistic regression analysis was used to present the adjusted odds ratio of having had an abortion in the last 5 years with the predictor variables controlling for other potential confounders. All analyses took into account the complex survey design. A *p*-value less than 0.05 was considered statistically significant.

## Results

Table 1 presents the number of abortions women of reproductive age had in the last 5 years. Overall, 4% (95% CI: 3.41–4.29) had had an induced abortion in the last 5 years, with less than 1% having had more than one induced abortion (data not shown in the table). Higher proportions of induced abortion were observed among women who were aged 20–34 years (5.7%) compared to women aged below 20 years and 35–49 years, had primary level education (5.1%), were from the richest wealth quintile (5.4%), had one living male child already (5.5%), and knew abortion is legal (5.5%). The lowest proportions were observed among women who reside in Province 2 (2.4%) and belong to specific ethnic groups (Terai Dalit (2.1%), Terai Janajati (1.6%), and Muslims (2.4%)). No significant differences in induced abortion were observed by place of residence or ecological zone.

Table 2 presents the unadjusted and adjusted odds ratios (AORs) of women of reproductive age who have had an induced abortion in the last 5 years associated with selected background characteristics. The AOR of induced abortion was significantly higher among women aged 20–34 years (AOR: 5.54; 95% CI: 2.87–10.72) compared to women aged < 20 years and among women educated through primary level only (AOR: 1.35; 95% CI: 1.02–1.79) compared to women having no education. Likewise, compared to women who reside in Province 1, higher odds of induced abortion were observed among women who reside in Province 4 (AOR: 1.56; 95% CI: 1.04–2.34), Province 5 (AOR: 1.66; 95% CI: 1.11–2.49), Province 6 (AOR: 2.10; 95% CI: 1.30–3.39) and Province 7 (AOR: 1.75; 95% CI: 1.14–2.69).

**Table 1:** Characteristics of women of reproductive age who had an induced abortion in the last 5 years (*n* = 12,862)

	Induced Abortion Care Received			Number of Women
	n	%	95% CI	
Age (years)^a^				
< 20	19	0.7	0.04–1.73	2598
20–34	354	5.7	5.02–6.50	6192
35–44	119	2.9	2.39–3.59	4072
Education^a^				
No education	133	3.1	2.54–3.79	4281
Primary	109	5.1	4.04–6.31	2150
Secondary	186	4.1	3.48–4.89	4516
Higher	64	3.4	2.53–4.43	1915
Residence				
Urban	336	4.2	3.62–4.78	8072
Rural	156	3.3	2.65–4.00	4790
Province^a^				
Province 1	67	3.1	2.19–4.33	2173
Province 2	60	2.4	1.72–3.22	2564
Province 3	92	3.4	2.41–4.66	2733
Province 4	68	5.4	4.44–4.66	1249
Province 5	106	4.7	3.66–5.97	2274
Province 6	41	5.7	4.21–7.56	724
Province 7	58	5.0	3.87–6.50	1145
Ecological zone				
Mountain	33	4.2	2.65–6.59	775
Hill	235	4.2	3.60–4.99	5556
Terai	224	3.4	2.88–4.08	6531
Wealth quintile^a^				
Poorest	69	3.2	2.35–4.25	2176
Poorer	82	3.2	2.54–4.14	2525
Middle	87	3.3	2.70–4.12	2595
Richer	103	3.8	3.02–4.65	2765
Richest	151	5.4	4.49–6.47	2801
Aware of abortion legalization^a^				
No	137	2.6	2.06–3.14	5362
Yes	287	5.5	4.74–6.36	5224
Don’t know	68	3.0	2.36–3.84	2276
Number of living children^a^				
0–1	153	2.6	2.10–3.20	5901
2	149	5.0	4.11–6.00	3007
3+	190	4.8	4.03–5.71	3954
Living boy child^a^				
0	125	2.3	1.9–2.9	5352
1	230	5.5	4.8–6.4	4145
2	108	4.3	3.5–5.3	2523
3+	29	3.5	2.4–5.0	842
Caste/ethnicity^a^				
Hill Dalit	66	6.3	4.95–8.02	1042
Terai Dalit	11	2.1	1.13–3.78	554
Hill Brahmin	69	4.6	3.52–5.89	1512
Hill Chhetri	118	5.0	4.10–6.12	2344
Terai Brahmin/Chhetri	7	3.3	1.36–7.66	217
Other Terai caste	59	3.1	2.27–4.16	1908
Newar	27	4.2	2.27–7.58	639
Hill Janajati	100	3.7	2.97–4.66	2694
Terai Janajati	20	1.6	0.99–2.61	1266
Muslim	15	2.4	1.40–3.90	643
Other	0	0.0	–	43
Total	492	3.8	3.41–4.29	12,862

^a^Statistically significant confidence interval

**Table 2:** Bivariate and adjusted associations between induced abortion in the past 5 years and potential correlates (*n* = 12,862)

	Bivariate Analysis			Multivariate Analysis^a^		
	OR	95% CI	P	AOR	95% CI	P
Age (years)						
< 20	1			1		
20–34	8.22	4.46–15.14	< 0.001	5.54	2.87–10.72	< 0.001
35–44	4.10	2.16–7.78	< 0.001	1.94	0.93–4.04	0.076
Education						
No education	1			1		
Primary	1.66	1.27–2.18	< 0.001	1.35	1.02–1.79	0.037
Secondary	1.34	1.03–1.75	0.031	1.25	0.90–1.72	0.181
Higher	1.08	0.75–1.57	0.667	0.68	0.44–1.05	0.080
Residence						
Urban	1			1		
Rural	0.77	0.60–1.00	0.053	0.92	0.71–1.19	0.523
Province						
Province 1	1			1		
Province 2	0.76	0.47–1.22	0.254	0.89	0.48–1.62	0.701
Province 3	1.09	0.67–1.78	0.729	0.88	0.53–1.42	0.577
Province 4	1.81	1.20–2.73	0.005	1.56	1.04–2.34	0.031
Province 5	1.54	1.00–2.38	0.052	1.66	1.11–2.49	0.014
Province 6	1.88	1.18–3.01	0.008	2.10	1.30–3.39	0.003
Province 7	1.66	1.06–2.59	0.026	1.75	1.14–2.69	0.010
Ecological zone						
Mountain	1			1		
Hill	1.01	0.61–1.68	0.966	0.99	0.94–2.04	0.971
Terai	0.81	0.49–1.35	0.419	1.00	0.56–1.78	0.991
Wealth quintile						
Poorest	1			1		
Poorer	1.03	0.70–1.49	0.896	1.39	0.94–2.05	0.099
Middle	1.06	0.73–1.53	0.770	1.62	1.08–2.43	0.020
Richer	1.19	0.82–1.73	0.357	1.74	1.16–2.62	0.008
Richest	1.74	1.21–2.50	0.003	2.80	1.79–4.39	< 0.001
Aware of abortion legalization						
No	1			1		
Yes	2.22	1.71–2.90	< 0.001	2.28	1.77–2.94	< 0.001
Don’t know	1.19	0.87–1.63	0.285	1.25	0.91–1.73	0.175
Number of living children						
0–1	1			1		
2	1.97	1.45–2.67	< 0.001	1.24	0.83–1.86	0.282
3+	1.90	1.44–2.49	< 0.001	2.24	1.51–3.31	< 0.001
Living boy child						
0	1			1		
1	2.44	1.92–3.12	< 0.001	1.50	1.07–2.09	0.018
2	1.86	1,40–2.48	< 0.001	1,22	0.81–1.84	0.339
3+	1.51	1.00–2.27	0.05	1,10	0.64–1.91	0.727
Caste/ethnicity						
Hill Dalit	1			1		
Terai Dalit	0.31	0.16–0.62	0.001	0.40	0.18–0.93	0.033
Hill Brahmin	0.71	0.49–1.03	0.073	0.62	0.39–0.99	0.045
Hill Chhetri	0.78	0.57–1.07	0.123	0.73	0.52–1.03	0.079
Terai Brahmin/Chhetri	0.50	0.20–1.27	0.146	0.47	0.16–1.32	0.151
Other Terai caste	0.47	0.31–0.71	< 0.001	0.48	0.27–0.83	0.010
Newar	0.65	0.34–1.25	0.193	0.82	0.46–1.69	0.582
Hill Janajati	0.57	0.41–0.80	0.001	0.67	0.46–0.96	0.028
Terai Janajati	0.24	0.14–0.43	< 0.001	0.24	0.13–0.47	< 0.001
Muslim	0.36	0.20–0.64	0.001	0.41	0.21–0.81	0.010

^a^Adjusted odds ratio has been adjusted for all variables listed

Moreover, women in the richest wealth quintile had almost three times the odds of having had an induced abortion in the last 5 years (AOR: 2.80; 95% CI: 1.79–4.39) when compared with those in the poorest wealth quintile, and the odds of induced abortion increased with each category in wealth quintile. Higher odds of induced abortion were observed among women who have knowledge about abortion legalization (AOR: 2.28, 95% CI: 1.77–2.94) compared to those who think abortion is not legal in Nepal. Also, a strong association was observed among the number of living children and an induced abortion in the last 5 years. Women with a higher number of living children had higher odds of seeking induced abortion services. Compared to those having no living boy child, women having one living boy child had higher odds of seeking induced abortion services (AOR: 1.50, 95% CI: 1.07–2.09). However, no association was observed between induced abortion services and those having two or more than two living male children.

Compared to Hill Dalits, lower odds of an induced abortion were observed among Terai Dalits (AOR: 0.40; 95% CI: 0.18–0.93), Hill Brahmin (AOR: 0.62, 95% CI: 0.39–0.99), Hill Janajatis (AOR: 0.67; 95% CI: 0.46–0.96), Terai Janajatis (AOR: 0.24; 95% CI: 0.13–0.47), Muslims (AOR: 0.41; 95% CI: 0.21–0.81) and other Terai caste (AOR: 0.48; 95% CI: 0.27–0.83).

## Discussion

This sub-analysis of data yielded by a nationally representative survey assesses induced abortion among women of reproductive age and its correlates. Overall, less than 4% of women of reproductive age had an induced abortion in the 5 years preceding the survey, and less than 1% had more than one induced abortion. The study found that the proportion of women who reported an induced abortion varied greatly by socio-demographic characteristics, economic status, and knowledge on abortion legalization. Women aged 20-34 years, urban dwellers, residents of Province 6, those in the richest wealth quintile, and women who know abortion is legal were more likely to have had an abortion in the last 5 years. Additionally, the highest proportion of women who reported an induced abortion was observed among Hill Dalits, whereas the lowest proportions were among ethnic communities of Terai, Janjati, Dalits, and Muslims.

We found that induced abortion was highest among the age group 20–34 years. However, there is not a specific pattern in abortion by age as previously observed in other countries. A study from Sweden reported a U-shaped pattern with age (that is, it is highest for the youngest and for oldest age groups). A study from Tehran found that abortion rates peaked among those aged 20–34 years, which is consistent with this study [24, 25]. A possible reason is that women aged 20–34 years are generally engaged in work and do not want child bearing to conflict with their career growth [26]. Despite frequent media reports that induced abortion is being used as a contraceptive method in Nepal and that a considerable proportion of women are having multiple induced abortions, the evidence from our study does not show this. Our findings show that less than 4% of women of reproductive age had an induced abortion in the last 5 years and that far fewer (less than 1%) had more than one induced abortion. Moreover, among women who had had an induced abortion in the last 5 years, only 13% reported multiple abortions.

Evidence from elsewhere suggests that women whose youngest living child is female are more likely to seek an induced abortion, thus linking induced abortion service with sex selection [27, 28]. Although 6.5% of respondents interviewed in the Nepal 2016 Demographic Health Survey reported sex of the child as their reason for an induced abortion [10], no statistical association was observed between induced abortion in the last 5 years and those who don’t have a living boy child. In fact, the likelihood of seeking abortion services was significantly higher among those who had at least one living boy child. The findings might infer either the tendency to have both son and daughter in the family or the likelihood of seeking induced abortion services due to unintended pregnancies. This study revealed a strong association between induced abortion and number of living children. This implies women who have achieved desired fertility but conceived due to non-use or inconsistent use of contraceptives or those who experienced contraceptive failure resort to abortion services. Similar associations were reported in other studies [14, 29].

The overall disparities in induced abortion utilization in relation to different socio-economic strata should be considered in the context of health inequities in Nepal and why certain groups are left behind in utilizing health care services [30]. There is a gap in health service utilization based on ethnicity, wealth status, education status, ecology, place of residence and provinces [31, 32]. The province level disparities may be attributed to poor health infrastructure, disparities in wealth status and caste/ethnicity make up of the provinces. Moreover, provincial-level disparities are of importance as Nepal has recently transitioned to a new federal structure with seven provinces, and our paper provides province-wise data that can help to roll out safe abortion programs at the province level.

This study also revealed a positive association between wealth quintile and induced abortion [33]. Wealth status determines the purchasing capacity for health care services, and at the time the 2016 NDHS survey was conducted, abortion care services were not free of charge and poor women may have faced cost barriers. Beside procedure cost, other indirect costs such as transportation might impede women as abortion care services are not widely accessible throughout Nepal [17]. There was also substantial ethnic variation in induced abortion utilization. Muslims and Terai Dalits had significantly lower odds of having had an induced abortion even though their unmet need for family planning is high [30], suggesting that these groups lack access to reproductive health services more broadly. Similar to other reproductive health services, women’s autonomy, awareness, cultural and religious beliefs, and cost can be potential factors that lead to lower rates of induced abortion among these groups [34–36].

The strength of this study is that it is based on a large, nationally representative sample consisting of both urban and rural populations, with a high response rate of 98%. However, the study’s findings should be viewed in light of its limitations. As with other cross-sectional studies, a causal relationship cannot be established. In addition, another limitation is the sensitive nature of the primary outcome of induced abortion, which might have led to it being under reported [37]. To minimize this, the questionnaire was designed in such a way to account for all pregnancies and the outcome of each pregnancy. Confidentiality and anonymity of the responses were assured to respondents throughout the survey.

## Conclusions

The findings of this study help fill the evidence gap on induced abortion and its correlates in Nepal. We found that abortion utilization is correlated with women’s age, knowledge on abortion legalization, wealth status, number of living children, and ethnicity. We recommend that the health system and administrators put extra effort into strengthening contraceptive provision and abortion education programs, and to improving access to abortion services for disadvantaged groups. In addition, we recommend further study to explore the reasons behind the ethnic variations in induced abortion in Nepal.
